The article "Bioengineering of anaerobic digestion for volatile fatty acids, hydrogen or methane production: A critical review" was retracted in 2026. Reason: compromised peer review.

# Bioengineering of anaerobic digestion for volatile fatty acids, hydrogen or methane production: A critical review

**DOI:** 10.1080/21655979.2019.1673937

**Published:** 2019-10-13

**Authors:** Steven Wainaina, Lukitawesa, Mukesh Kumar Awasthi, Mohammad J. Taherzadeh

**Affiliations:** a Swedish Centre for Resource Recovery, University of Borås, Borås, Sweden; b College of Natural Resources and Environment, Northwest A&F University, Yangling, Shaanxi Province, PR China

**Keywords:** Anaerobic digestion, metabolic pathways, volatile fatty acids, hydrogen, biorefineries, process parameters, mixed culture fermentation, inhibiting methanogens

## Abstract

Anaerobic digestion (AD) is a well-established technology used for producing biogas or biomethane alongside the slurry used as biofertilizer. However, using a variety of wastes and residuals as substrate and mixed cultures in the bioreactor makes AD as one of the most complicated biochemical processes employing hydrolytic, acidogenic, hydrogen-producing, acetate-forming bacteria as well as acetoclastic and hydrogenoclastic methanogens. Hydrogen and volatile fatty acids (VFAs) including acetic, propionic, isobutyric, butyric, isovaleric, valeric and caproic acid and other carboxylic acids such as succinic and lactic acids are formed as intermediate products. As these acids are important precursors for various industries as mixed or purified chemicals, the AD process can be bioengineered to produce VFAs alongside hydrogen and therefore biogas plants can become biorefineries. The current review paper provides the theory and means to produce and accumulate VFAs and hydrogen, inhibit their conversion to methane and to extract them as the final products. The effects of pretreatment, pH, temperature, hydraulic retention time (HRT), organic loading rate (OLR), chemical methane inhibitions, and heat shocking of the inoculum on VFAs accumulation, hydrogen production, VFAs composition, and the microbial community were discussed. Furthermore, this paper highlights the possible techniques for recovery of VFAs from the fermentation media in order to minimize product inhibition as well as to supply the carboxylates for downstream procedures.

## 1. Introduction

The growing global population has led to an increase in the amounts of organic wastes that require appropriate treatment. Relative to other treatment methods, such as composting, incineration and landfilling, anaerobic digestion has been widely accepted as a flexible and eco-friendly treatment method that not only stabilizes these wastes but also provides an avenue for energy recovery [1,2]. Naturally-occurring microbial communities are involved in the breakdown of organic matter in several successive and inter-dependent stages resulting in biogas that is rich in methane. Biogas is generally used for generation of heat and electricity as well as a transport fuel. Research in the application of the anaerobic digestion process is increasingly shifting to other intermediate metabolites of higher value than biogas that includes hydrogen and carboxylic acids such as lactic, succinic and volatile fatty acids (VFAs) [3]. The VFAs are carboxylates with low molecular weight consisting of 2 to 6 carbon atoms with properties provided in Table 1 and are conventionally derived from petroleum. Besides being precursors to the production of biodegradable plastics and biofuels, VFAs can be used for removal of nitrogen and phosphorus during wastewater treatment and can also converted into a wide array of bio-chemicals that are essential for several manufacturing industries (Table 1) [4]. The bio-synthesis of VFAs from wastes could therefore potentially transform anaerobic digestion facilities into biorefineries. Some of the organic residues explored for production of VFAs include food waste [4], lignocellulosic biomass [5], waste activated sludge [6], wastes from fish processing industries [7], cassava wastewater [8], pulp and paper mill as well as dairy whey effluents [9].

The article "Bioengineering of anaerobic digestion for volatile fatty acids, hydrogen or methane production: A critical review" was retracted in 2026. Reason: compromised peer review.

**Table 1.** Physicochemical properties and potential applications of individual volatile fatty acids.

VFA	Molecular formula	Molecular weight (g/mol)	Boiling point (°C)	pKa	Area of application
Acetic	CH_3_COOH	60.05	118	4.76	Food additives, plasticizers, dyes
Propionic	CH_3_CH_2_COOH	74.08	141	4.88	Resins, pharmaceuticals, paints
Isobutyric	(CH_3_)_2_CHCOOH	88.11	154	4.84	Pesticides, food additives, paints
Butyric	CH_3_CH_2_CH_2_COOH	88.11	164	4.82	Perfumes, textiles, vanishes, plastics
Isovaleric	(CH_3_)_2_CHCH_2_COOH	102.13	177	4.77	Pharmaceuticals, perfumes, fungicides
Valeric	CH_3_(CH_2_)_3_COOH	102.13	185	4.84	Perfumes, plasticizers, lubricants
Caproic	CH_3_(CH_2_)_4_COOH	116.16	205	4.88	Rubber, grease, tobacco flavor

Anaerobic digestion (AD) for production of renewable energy in the form of biogas or biomethane and even hydrogen, through the so-called dark fermentation, is well documented in the literature and there are several good reviews on these topics [10–12]. AD can generally be considered as a three-phase process that entails; (1) the breakdown of complex organic matter in the raw substrate into soluble substances, (2) the formation of VFAs and hydrogen and (3) the consumption of the VFAs and hydrogen for biogas production. The substrate solubilization utilizes hydrolytic bacteria such as *Acetivibrio Cellulolyiticus, Bacillus, Peptococcus*, and *Vibrio* [13]. For organic wastes with recalcitrant structure, an initial pretreatment prior to the anaerobic biodegradation is needed [14]. After hydrolysis, fast-growing acidogens and acetogens, such as *Butyribacterium* and *Clostridium*, rapidly convert the soluble substances into VFAs [11,13,15]. It is also possible to design the process such that hydrogen is metabolized as the main product from the biodegradation of the wastes. The hydrogen production during the acidification step is also referred to as dark fermentation to distinguish it from other microbial processes such as photofermentation and biophotolysis [12,16]. The buildup of VFAs in the bioreactors should be balanced with suitable extraction strategies to circumvent potential product inhibition on the cells as well as to supply the carboxylic acids for further processing or application [17]. Finally, the hydrogen- and VFAs-consuming methanogens in the microbial consortium should be selectively deactivated [4]. Several authors have investigated the influence of physicochemical parameters on the above-mentioned phases, such as pH, temperature, organic loading rate (OLR), hydraulic retention time (HRT) and substrate pretreatment [9,18–21]. A few reports have also proposed the possible acidogenic biological pathways that lead to a varied distribution of the VFAs, mainly as a function of pH [22,23]. However, the biochemistry and engineering aspects for sustained high yields of VFAs and hydrogen from wastes, considering the above broad phases, have not yet been systematically described in literature.

The article "Bioengineering of anaerobic digestion for volatile fatty acids, hydrogen or methane production: A critical review" was retracted in 2026. Reason: compromised peer review.

Therefore, the goals of this review were to: (1) provide the microbial and kinetic characteristics contributing to the production, distribution and accumulation of VFAs, (2) explain the substrate-related issues that require attention prior to the bio-conversion process, (3) describe the possible methods of manipulating the AD process toward production of more or less hydrogen relative to VFAs, (4) elucidate the potential methods of preventing the conversion of VFAs and hydrogen into biogas and, (5) propose sustainable VFAs recovery techniques.

## 2. Microbial production of particular VFAs and hydrogen using pure cultures

The conventional route for industrial production of the individual VFAs depends on petroleum-based chemicals. As an alternative production route, several natural and modified microorganisms that utilize bio-based substrates have been explored. Acetic acid, for instance, can be produced via chemical catalytic reactions from methanol and ethylene [24]. Various kinds of microbes, such as *Thermoanaerobacter, Acetomicrobium*, and *Clostridium*, can be used for acetic acid production via the fermentation route. Notably, *Acetobacter* and *Gluconobacter* have been commercially applied [25,26]. In order to enhance productivity, operating parameters have been optimized to convert distinct kinds of sugars (such as glucose, melibiose and arabinose) into acetate [27]. Finding novel carbon source alternatives and integrated processes is however critical due to higher economic cost of the commercial sugars. Application of biomass such as lignocellulose and cellulose as potential alternates was found to produce 17 g/L and 30.98 g/L acetic acid by *Clostridium lentocellum*, respectively [28].

The article "Bioengineering of anaerobic digestion for volatile fatty acids, hydrogen or methane production: A critical review" was retracted in 2026. Reason: compromised peer review.

Propionic acid is a significant carboxylate at a compound annual growth rate of 2.7% of 470.0 kilotons by 2020 [29]. Most of the propionic acid bacteria belong to the genus *Propionibacterium*, including *P. freudenreichii, P. acidipropionici, P. thoenii, P. shermanii*, and *P. jensenii* [30]. The productivity of propionic acid reached 0.71 g/g by use of glycerol that was a more cost-effective material than commercial sugars compared to glucose was 0.35 g/g [31]. Furthermore, utilization of low-cost cane molasses by *P. acidipropionici* action could generate 30 g/L propionic acid [32]. In addition, genome shuffling technology could increase 25% of *P. acidipropionici* [33]. Moreover, the production of propionic acid reached at 26.95 g/L and 34.93 g/L by the action of engineered *P. jenseniis* [34].

Butyric acid is also a valuable commodity with a projected demand of 105 kilotons by 2020 [29,35]. Generally, butyric acid can be produced by butyraldehyde oxidation from crude oil as well as through fermentation [36]. Various kinds of microbial strains contribute to butyric acid production during fermentation, such as *Clostridium barkeri, C. thermobutyricum, Butyribacterium* sp., *Fusobacterium nucleatum, Butyrivibrio fibrisolvens, Sarcina* and *Eubacterium limosum* [29]. Fermentation with *Clostridium tyrobutyricum* has previously shown a 0.37–0.46 g/g butyrate productivity with glucose together with xylose yielding up to 34.2 g/L butyric acid [37]. Very high production of butyric acid from glucose (up to 86.9 g/L) was achieved by a fed-batch fermentation strategy in a fibrous bed bioreactor with immobilized *Clostridium tyrobutyricum* [38]. Genetic engineering technique was also employed with some non-producer bacterial strains such as *Escherichia coli*, to generate butyrate by excluding major NADH-dependent oxidation/reduction process, re-hypothesizing the metabolic pathway for butyryl-CoA, and overexpressing *ato* AD genes as a requisite to transform butyryl-CoA to butyrate and withdrawing acetate-synthesis pathways. Thus, Saini et al. [39] developed an *E. coli* strain to generate 10 g/L butyrate from the beginning of process and conversion of glucose to acetate as carbon source.

The article "Bioengineering of anaerobic digestion for volatile fatty acids, hydrogen or methane production: A critical review" was retracted in 2026. Reason: compromised peer review.

Isovalerate can chemically be produced by oxidation of isoamyl alcohol and biologically from *Propionibacterium freudenreichii* [40]. Zhang et al. [41] reported 11.7 g/L production of isobutyrate under the action of engineered *E. coli* during glucose fermentation. Regarding production of isovaleric acid, Xiong et al. [42] found a concentration of up to 32 g/L would be produced using an engineered *E. coli* strain. Lang et al. [43] also found that a genetically modified strain, *Pseudomonas* sp. strain VLB120, used valine degradation pathway to generate only 2.3 g/L isobutyric acid via isobutyryl-CoA.

Pure cultures have also been extensively studied for the production of bio-based hydrogen. For example, one research was carried using *Bacillus coagulans* in which 2.28 mol hydrogen/mol glucose at 37°C and pH 6.5 was attained [44]. In another report, *Clostridium pasteurianum* was applied resulting in the highest hydrogen production at pH 6.0 and a yield of up to 2.33 mol hydrogen/mol glucose [45]. On the other hand, *Enterobacter cloacae* was found to produce 2.25 mol hydrogen/mol glucose optimally at 36°C [46]. Sucrose showed the best production rate at 660 mol hydrogen/L/h at pH 6.0, which was a better performance compared to L-arabinose, D-xylose, glucose, cellobiose, and fructose [46]. Lastly, the optimal pH ranges using a novel *Clostridium amygdalinum* strain were found to be 7.5–8.5 for xylose and pH 8.5 for arabinose which yielded 2.2–2.5 mol hydrogen/mol substrate and 1.78 mol hydrogen/mol substrate, respectively [47].

### 2.1. Production of VFAs from organic wastes

The biotechnological processes explained in the previous section use pure cultures that can be optimized for specific strains of microorganism [48]. For the last few decades, researchers have explored different means to produce VFAs through fermentation by utilizing a range of carbon sources as raw materials [49–52]. Most VFAs production is based on using pure sugars and such processes lead to higher productivity with minimum side products [52–54]. However, the advantage of higher productivity and yield of such processes may be negated by the higher cost of the raw materials. It is worth mentioning that besides VFAs, acidogenic fermentation of wastes can also yield other high-value products based on the established metabolic pathways [55]. These metabolites can be obtained as by-products in low concentrations and include succinate, ethanol and isopropanol [23,56]. Lactic acid can also be synthesized in acidification bioreactors enriched with microbes such as *Clostridium, Dysgonomonas*, and *Streptococcus* [57].

The article "Bioengineering of anaerobic digestion for volatile fatty acids, hydrogen or methane production: A critical review" was retracted in 2026. Reason: compromised peer review.

To reduce production costs, researchers are now focusing on using abundantly available lignocellulose biomass as a carbon source for VFAs production [58,59]. Microorganisms are not able to directly utilize complex lignocellulose biomass, so the biomass must be pretreated using various physical, chemical, and enzymatic methods, thus adding to the process cost [60–62]. Moreover, applying pure cultures has fundamental disadvantages which include the requirements of sterile operating conditions and high-quality (and very often, high-purity) raw material. Mixed culture fermentation, on the other hand, does not rely on specific microorganism’s strain and can be operated in non-sterile conditions without significant risk of contamination [48,63]. Moreover, mixed culture fermentation is able to consume a broad spectrum of substrates containing diverse organic chemical compounds. Due to those characteristics, this type of fermentation can be fed with municipal, agricultural, or industrial waste streams [64] so that it does not have to use human-food resources. The mentioned waste streams are produced in vast amounts and their utilization into useful products would bring significant advantages. First of all, it would decrease the amount of waste generated; secondly, it would provide sustainable products (in contrast to fossil-based product) while cutting down the of emission greenhouse gases. If optimized, mixed culture fermentation processes have a great chance to outcompete pure culture fermentations.

### 2.2. Overview of the anaerobic digestion process

Anaerobic digestion (AD), the best example of mixed culture fermentation, is a biological process where most organic matter except for lignin components, in the absence of oxygen, is degraded into a final product consisting mainly of methane and carbon dioxide. The process consists of a series of reactions, and it is a natural process which takes places in several anaerobic environments [65,66]. Typically, AD provides a renewable energy source (biomethane), and it also delivers highly efficient natural fertilizer. Biological conversion such as AD that converts wet biomass waste into biogas is a well-established technology [67], whereas conversion of biomass waste to high-value biochemicals such as VFAs is mainly in the initial research phase [68–70].

Anaerobic digestion is a sequential process wherein hydrolysis is the first step, followed by acidogenesis, acetogenesis, and methanogenesis. These steps are achieved by the action and syntrophic association of various bacteria viz. hydrolytic, acidogenic, hydrogen-producing, acetate-forming microbes as well as acetoclastic and hydrogenoclastic methanogens [71]. Each stage of anaerobic digestion yields important bio-products: hydrolysis yields dissolved molecules such as fermented sugars and amino acids, acidogenesis yields VFAs and hydrogen, acetogenesis yield acetic acid and hydrogen while the final process, methanogenesis, yields mainly methane and carbon dioxide (biogas) [72]. During hydrolysis, complex organic polymers in waste are cracked down into simpler organic monomers by the enzymes excreted from the hydrolytic microorganisms. Then, acidogens ferment these monomers into pyruvic acid through various pathways such as the Embden-Meyerhof pathway, and pentose phosphate pathway, Bifidus pathway. On the other hand, through the Entner-Doudoroff pathway and phosphoketolase pathway, ethanol, and lactate are produced [22]. In those processes, a complex consortium of obligate and facultative anaerobes are involved, such as *Clostridia, Bacteriocides, Bifidobacteria, Enterobacteriaceae*, and *Streptococci* [73]. However, most of the anaerobic bioreactors conduct the hydrolysis and acidogenesis process simultaneously in a single bioreactor.

The article "Bioengineering of anaerobic digestion for volatile fatty acids, hydrogen or methane production: A critical review" was retracted in 2026. Reason: compromised peer review.

Hydrogen production during the acidification step is also referred to as dark fermentation and is catalyzed by either facultative or strict anaerobes and even some aerobes [16]. The specific catabolic processes involved in hydrogen production are well explained in literature [74,75]. The dark fermentation processes have been carried out using inocula from sources such as sludge from a dairy farm digester and palm oil mill effluent as well as anaerobic sludge from municipal wastewater plants. Microbes responsible for hydrogen production under mesophilic conditions include *Clostridium butyricum, Clostridium pasteurianum, Clostridium saccharobutylicum* and *Enterobacter aerogenes* while in thermophilic conditions, *Caldicellulosiruptor saccharolyticus* and *Thermoanaerobacterium thermosaccharolyticum* have been identified [11]. Regarding the metabolic pathways toward hydrogen production, the so-called acetate and butyrate pathways are involved in carbohydrates fermentation and are capable of yielding a maximum of 4 and 2 mol hydrogen per mol of glucose, respectively [55].

The last phase of the anaerobic digestion is dominated by a particular group of microorganisms, which is called the methanogenic archaea. These are characterized through the co-factor F_420_, which acts in the presence of hydrogenase as a carrier for hydrogen, appears only in methanogens. Active methanogens appear in the second phase of fermentation, the acidogenic phase, but the number of methanogenic archaea increases in the methanogenic phase. *Methanobacterium, Methanospirillum* and *Methanosarcina* are some of the methanogenic genera involved in biogas production [76].

The article "Bioengineering of anaerobic digestion for volatile fatty acids, hydrogen or methane production: A critical review" was retracted in 2026. Reason: compromised peer review.

## 3. Theory of microbial synthesis of VFAs from organic wastes

Overall, dedicated VFAs bioprocesses using organic wastes as substrates are dependent on techniques to boost the substrates’ solubilization and consequent acidification while suppressing the consumption of the acids. For complex substrates that are difficult to biodegrade, the solubilization can be accelerated through an initial pretreatment process, among other options. For enhanced acidification, certain conditions are induced to ensure optimum microbial activities as well as manipulating the metabolic pathways suitable for synthesizing the desired end product. Finally, the methanogenic phase should be inhibited as much as possible and this can be achieved using chemicals, physicochemical parameters, or the application of heat. The various techniques applied for the substrate preparation, acidogenesis and inhibition of methanogen will be the focus of discussion in the subsequent sections.

The anaerobic digestion process involves a series of interdependent biochemical reactions. These reactions, summarized in Figure 1, are mainly controlled by the process rate-kinetics and physicochemical operating parameters [77–79]. The hydrolysis process occurs in the first phase and has been widely accepted to be the rate-limiting step that follows single first-order kinetics defined in equation 1 [80,81]. Some of the first-order constants reported in literature using mixed bacterial cultures are provided in Table 2. This first phase involves hydrolytic bacteria either attaching to the surface of the organic matter particles where the hydrolases are released or by first discharging the enzymes to the bulk medium from where they attack the organic particles. During the hydrolytic reactions, the macromolecules in the form of carbohydrates, lipids and proteins are broken down into monosaccharides, long-chain fatty acids, and amino acids, respectively, that can easily pass through the cell membrane [80–82]. For recalcitrant materials and other complex organic wastes, an extra disintegration process is necessary, either as a prior process or even during fermentation [14,83].

(1) $$F=\frac{F_{0}}{1+k_{h}\theta }$$

**Table 2.** First-order hydrolysis constants for selected macromolecules in organic wastes [81].

Substrate	T (°C)	First-order rate constant (day ^−1^)	Mode of cultivation
Starch	35	0.20–1.08	Semi-continuous
Cellulose	35	0.12	Batch
Cellulose	35	0.28–0.52	Semi-continuous
Glutamic acid	35	1.12	Semi-continuous
Leucine	35	0.31–0.63	Semi-continuous
Gelatin	37	0.60	Batch

The article "Bioengineering of anaerobic digestion for volatile fatty acids, hydrogen or methane production: A critical review" was retracted in 2026. Reason: compromised peer review.

**Figure 1.** Schematic flow of the reactions involved in formation of volatile fatty acids coupled with the product extraction during anaerobic digestion.

where *F* = final concentration of degradable organics, *F_0_* = initial concentration of degradable organics, *k_h_ *= degradation rate constant and θ = hydraulic retention time.

The products of hydrolysis are then consumed by acidogens and acetogens which metabolize mainly VFAs and hydrogen, as well as other by-products such as carbon dioxide and alcohols [84]. The growth kinetics of the acid-forming bacteria can be summarized by the relationship in Equation 2 [74]. Acidogens, which are responsible for the initial degradation reactions of the hydrolyzed compounds, require short durations of doubling time depending on the available bacteria and the specific compound [75,81]. Some growth coefficients and doubling times during the acid-forming phase are provided in Table 3. In general, the estimated minimum retention time between 1–2 days is needed for completing the reactions leading to biosynthesis of VFAs [77]. The accumulation of VFAs that occurs in the second phase can result in a sharp drop in pH levels and the VFAs exist mainly as undissociated acids at pH levels below the acids’ dissociation constant (≤ 4.86 at 25 °C) [85]. These undissociated acid molecules can easily diffuse into the cell’s cytoplasm resulting in microbial inhibition [86,87]. As a result, appropriate techniques are required to continually extract the metabolized acids from the bioreactor, as indicated in Figure 1. Moreover, this extraction can also aid in recovery of the VFAs for further processing or direct application.

(2) $$r_{s}=\frac{1}{Y_{X/S}}.\frac{\mu_{max}.S}{K_{S}+S}.X-b.X$$

**Table 3.** Typical kinetic constants during acidogenesis of hydrolysis products [74,81].

Substrate	µ*_max_* (day^−1^)	Y*_X/S_* (mg VSS/mg COD)	K*_S_* (mg COD/L)	Doubling time (h)	b (day^−1^)
Glucose	1.25	0.162	22.5^a^	0.5	–
Glucose	0.3	0.15	400^a^	2.3	–
Cellulose	0.071	0.16	36.8^a^	9.8	–
Unsaturated oleic acid	0.44	0.11	3180	–	0.01
Unsaturated linoleic acid	0.55	0.11	1816	–	0.01
Saturated myristic acid	0.105	0.11	105	–	0.01
Saturated stearic acid	0.085	0.11	417	–	0.01

^a= reported as mg/L^

where *r_s_* = substrate consumption rate, Y*_X/S_* = biomass yield factor, µ*_max_ *= maximum specific growth rate, S = amount of substrate, K*_S_* = saturation constant, X = amount of biomass and *b* = specific decay rate.

## 4. Formation of hydrogen versus VFAs

The general similarities that exist between VFAs and hydrogen as metabolites of the anaerobic digestion process are that they are biosynthesized as intermediaries and serve as precursors of biogas production. Due to the potential of obtaining these metabolites from organic residues, many researchers have successfully limited the methanogens activities with the aim of optimizing the formation of either VFAs or hydrogen [17,88–90]. From these studies, it can be concluded that bioprocesses that are favorable for the formation of the VFAs at high yields usually produce the hydrogen gas as a by-product, and vice versa. Indeed, it has been observed that the presence of VFAs interferes with hydrogen production, either as a result of inhibition by undissociated acid molecules [86] or due to consumption of hydrogen by homoacetogens [11]. The dissolved metabolites detected in the fermentation medium during fermentation of hydrogen are mainly acetate and butyrate due to the established pathways mentioned earlier. On the other hand, other reduced metabolites such as propionate are associated with low hydrogen production [91]. Regarding the impact of hydrogen on VFAs, it has been suggested that increasing the hydrogen partial pressure in the bioreactor could possibly alter the product spectrum of the acids [92].

The article "Bioengineering of anaerobic digestion for volatile fatty acids, hydrogen or methane production: A critical review" was retracted in 2026. Reason: compromised peer review.

The metabolic pathways of pure cultures can be directly controlled in order to improve the hydrogen yield [93]. However, anaerobic bioreactors use a variety of microflora that is robust, cheap and readily available in nature. The seeding inocula in the bioreactors undoubtedly dictate the end-product portfolio due to the enriched microorganisms and available enzymes. In addition, some operational parameters play a substantial role in manipulating the microbial pathways and include the type of substrate, pH, and the applied temperature [11,16,86]. Unlike acid-forming microorganisms that are active in a broad range of pH values, the production of hydrogen in mixed culture systems seems to be limited within an optimal pH of 5.5 [94], with pH levels below 5.0 found to be inhibitory [90]. Regarding the type of preferred substrate, a higher biological hydrogen production potential has been realized with carbohydrate-rich materials relative to lipids and proteins [90,95]. The nature of the substrate also determines the production of VFAs [23] and also can divert the metabolic activity toward different VFAs. When it comes to the effect of temperature, mesophilic conditions (e.g 35°C) largely favor production of VFAs while hydrogen production seems to be enhanced by increasing the temperature levels [96–98]. One of the reasonable explanations is that in thermophilic conditions, e.g 60 and 75 °C, hydrogen-producing microorganisms such as *Clostridium thermocellum* and *Caldanaerobacter subterraneus* are more active [99].

However, it should be noted that due to the complexity of undefined mixed cultures, some of the appropriate parameters required for shifting the balance in favor of either metabolite might overlap. Furthermore, deviation from the above findings can be attributed to the interaction of other operating factors as observed by Wongthanate et al. [100]. Thus, prior to anaerobic degradation of organic residues aiming at optimum yields of either VFAs or hydrogen, screening tests are recommended.

The article "Bioengineering of anaerobic digestion for volatile fatty acids, hydrogen or methane production: A critical review" was retracted in 2026. Reason: compromised peer review.

## 5. Strategies to boost the production of VFAs

The concept of VFAs production is closely related in ruminants’ (e.g. cow) digestion system whereas complex organic substrates converted into VFAs. In the cow digestion system, the presence of methanogens is undesirable because they can convert VFAs into methane, which causes the ruminant to suffer bloating or flatulence [101]. The rule of thumb for maximizing the accumulation of VFAs is not only optimizing the production but also minimizing the consumption. Boosting production of VFAs can be done in different ways, depending on the substrate and the inoculum. Meanwhile, reducing consumption of VFAs can be done by appropriate methods for deactivating the methanogens such as inoculum pretreatment, overloading the system with the substrate so that high VFAs concentration can reduce the number of methanogens, or addition of certain chemicals that act as methanogen inhibitors.

### 5.1. The substrate-related issues for optimum VFAs production

The hydrolysis step during AD of lignocellulosic materials is often hindered by the hard-to-digest lignin structure and crystallinity of cellulose. These recalcitrant properties are often preventing the microorganisms from attacking the primary substrate cellulose (and hemicellulose) causing VFAs production relatively slow compared to less recalcitrant substrates such as food waste. Due to slow hydrolysis, the concentration of VFAs accumulated in the digestion system is usually too low to affect the methanogens’ activities. In order to improve hydrolysis, the lignocellulose material has to be pretreated to open the packed structure, remove the lignin, and change the crystalline cellulose into a more amorphous form. The pretreatment of lignocellulosic materials can be achieved either through either physical, chemical, or biological means [102].

Monomer-rich substrates can be rapidly converted into VFAs. Neutral pH can be more favorable for VFAs production from glucose compared to acidic and alkaline pH [89]. However, the presence of monomers can slow down the degradation of the solid fraction of the substrate due to product inhibition. Therefore, continuous removal of VFAs should be carried out to optimize the conversion of solid fraction. Substrates containing inhibitors, such as fruit waste, have been an issue during biogas production via the AD process. Several flavor compounds from fruits such as D-limonene, lactone, ketone, and phenolic, esters could reduce methane production [103–106]. VFAs production also seems to be inhibited by the presence of D-limonene in first stage digestion of citrus waste [107]. Essential oil, such as patchouli oil, also proved as reduce methane production [108]. Removal of D-limonene has been studied with the aim of improving methane production [106,109–111]. One of the studies applied solvent pretreatment using hexane to reduce the D-limonene content in orange peel. However, hexane residue also appeared to be an inhibitor in the anaerobic digestion process [111]. Although it remains unclear whether the solvent is only inhibiting methanogens or also hydrolysis, acidogens, and acetogens, generally, a solvent can be toxic for most of the microorganisms [112]. Future research could possibly identify the impact of the flavor compounds on the production of VFAs.

The article "Bioengineering of anaerobic digestion for volatile fatty acids, hydrogen or methane production: A critical review" was retracted in 2026. Reason: compromised peer review.

### 5.2. Process parameters for optimum production of VFAs

#### 5.2.1. pH level

Among the operational parameters, pH has a very strong effect on VFAs production from fermentation of food waste. Jiang et al. [113] studied the influence of different pH values, comprised of slightly acidic range (5.0–7.0), on VFAs production from synthetic kitchen waste. They found out that pH values between 6.0 and 7.0 brought an increase of approximately 20% in the hydrolysis rate, achieving up to 82 g/L soluble chemical oxygen demand (COD). At lower uncontrolled pH, the observed soluble COD was 60 g/L. This increase of solubilization allowed to double VFAs production in the batch bioreactor as a consequence of a higher hydrolytic enzymes activity and avoidance of inhibition due to acidification of the medium. Furthermore, a pH close to neutrality brought about a different distribution of VFAs, with butyric acid, acetic acid, and propionic acid accounting for approximately 50, 25, and 15% of total fermentation products respectively. Zhang et al. [114] investigated the effect of pH on fermentation performance in a bioreactor working in continuous mode, adjusting pH to a value of 5.0, 7.0, 9.0, and 11.0. This study confirmed that pH close to neutral leads to a better VFAs yield. In fact, at controlled pH of 7.0, fermentative metabolism was favored, and a VFAs yield of 0.27 gVFA/gTS (TS = total solids) was achieved compared to 0.15 gVFA/gTS in the control bioreactor, where the pH was not controlled. The positive effect of slightly acid-neutral conditions on microbial metabolism and therefore on fermentative production was demonstrated in another study in which, besides VFAs production, carbohydrates and proteins utilization rates were monitored. At pH set up at a value of 6.0, VFAs yield increased 7.5 times compared to pH 4.0 [4].

The article "Bioengineering of anaerobic digestion for volatile fatty acids, hydrogen or methane production: A critical review" was retracted in 2026. Reason: compromised peer review.

A study carried out by Dahiya et al. [115] emphasized the relationship between pH and individual VFAs obtained from acidogenic fermentation. They fermented food waste in bench-scale batch bioreactors, under the following conditions: temperature of 28°C, organic loading rate (OLR) of 15 kg COD/m^3^d and 10% inoculum. The pH was adjusted at the beginning of the experiment to 5.0, 6.0, 7.0, 8.0, 9.0, 10.0, and 11.0. The maximal total VFAs concentration was detected in the bioreactor operating with an initial pH of 10.0 (6.3 g/L), followed by pH 9.0 (5.17  g/L), pH 6.0 (4.5  g/L), pH 5.0 (4.2  g/L), pH 7.0 (4.1  g/L), pH 8.0 (3.8  g/L) and pH 11.0 (3.5  g/L). It must be taken into account that the consumption of the produced VFAs occurred for methane production. Therefore, it was not possible to conclude that alkaline pH was ideal for VFAs production as their concentrations were higher before their conversion. Concerning VFAs distribution pattern, pH 10.0 seemed to favor acetic acid production, which reached a maximal value of 4.2 g/L after 36 hours, after which it decreased up to approximately 3.6 g/L probably as a consequence of methane production. Butyric acid was the main fermentation product under a pH of 5.0 (1.8 g/L), and its concentration did not show a remarkable decrease between 36 and 48 hours. Propionic acid achieved a concentration of around 1.4 g/L under all pH values tested, and it was not consumed even after its maximal concentration was reached.

Overall, applying a pH level around 6.0 has been identified as suitable for enhanced production of VFAs from a variety of organic wastes [23]. Alkaline pH is also favorable for materials requiring an extensive hydrolysis process such as maize silage [89]. Controlling the pH is also an important factor because the production of VFAs can result in a sharp pH decrease. At pH levels below the dissociation constant (pKa) of VFAs, most of the acids are in undissociated form and can possibly harm the microorganisms.

#### 5.2.2. Organic loading rate (OLR)

Organic loading rate (OLR) indicates the amount of substrate fed into the bioreactor per day per unit of working volume, in terms of total solids (TS) volatile solids (VS) or COD. One important factor to be considered in operating at high OLR is the presence of inhibitors in the substrate. There are possibilities of the inhibitor affecting not only the methanogens but also the hydrolytic and acidifying bacteria. Lim et al. [98] studied the effect of OLR on acidogenesis, in a semi-continuous bioreactor. They observed that total VFAs production increased with an increase of OLR, achieving a maximum concentration of around 14.0, 24.0, and 30 g/L, with an OLR of 5.0, 9.0 and 13.0 gTS/L/d, respectively. Although the higher concentration at 13.0 g/Ld, the yield of VFAs was lower with respect to the lower OLR values, which could be ascribed to the high viscosity of the fermentation medium [98,116]. Among the three different OLRs tested (5.0, 9.0, and 11.0 gTS/L/d), an OLR of 9.0 gTS/L/d was most suitable for an appropriate VFAs production. A similar result was obtained from synthetic food waste fermented in semi-continuous bioreactors at 35 °C, pH 6.0, and hydraulic retention time (HRT) of 5 days. By an increment of OLR from 5.0 to 11.0 gTS/L/d, the total VFAs concentration increased from about 13.0 to 21.0 g/L. However, the yield was 13% better when an OLR of 5.0 gTS/Ld was adopted. It is important to remark that further increase of OLR from 11.0 to 16.0 gTS/Ld caused instability in the bioreactor, and a stable production rate was achieved by decreasing the OLR [113].

The article "Bioengineering of anaerobic digestion for volatile fatty acids, hydrogen or methane production: A critical review" was retracted in 2026. Reason: compromised peer review.

Another research by Gou et al. [117] examined a possible relationship between OLR and working temperature from a co-fermentation of waste activated sludge and food waste (mixed in a 2:1 ratio on TS basis) conducted in a semi-continuous mode. The OLR was increased from 1.0 to 8.0 gVS/L/d in three identical bioreactors operated at 35, 45, and 55 °C. They found out that a stable total VFAs of 4 g/L was achieved at higher temperature, while under mesophilic conditions the OLR must be kept under 5 gVS/L/d to obtain a stable total VFAs production of around 3.5 g/L. Therefore, the choice of an optimal OLR is fundamental in ensuring stable production of VFAs. To ensure a high product yield, the OLR should be abundant enough to provide an adequate amount of carbon-source to fermentative metabolism and also balanced with other operating conditions such as the applied temperature. In fact, under mesophilic conditions, an OLR higher than 5 gTS/L/d may cause the apparent viscosity increase of the fermentation medium, reducing the mass and heat transfers and consequentially the conversion of the substrate into VFAs.

#### 5.2.3. Temperature

Temperature is a crucial parameter during acidogenic fermentation, due to its direct involvement both in microbial growth and metabolism. Every microbial taxon has an optimum range of temperature for its replication. Consequently, a change of working temperature can alter the microbial structure of the microbial consortium involved in acidogenic fermentation. For instance, He et al. [118] found that an increase of operating temperature from mesophilic (35 °C) to thermophilic range (55 °C) brought to a decrease of total VFAs production from a maximum concentration of 17 g/L to 11 g/L. A further increase of temperature toward hyperthermophilic range (70 °C) caused a lower reduction of total VFAs production, which reached a maximum value of about 13 g/L. In another research by Komemoto et al. [119], the effect of temperature on acidogenic fermentation was explored between psychrophilic (15, 20 °C) and hyperthermophilic (65 °C) ranges. They found out that at 55 and 65 °C, the soluble sCOD in the bioreactor remarkably increased at the beginning of experiment up to a value of around 40 g/L, and afterward dropped quickly to 30 g/L. However, in the mesophilic range, the sCOD reached a similar value (30 g/L), but it remained stable until the end of the experiment. The difference was ascribed to microbial hydrolysis activity; at a higher temperature, solubilization is the result of a physicochemical effect, while in the mesophilic range, there is an active action of microbial enzymes. Concerning VFAs production, acetic acid was produced at the beginning of the experiment, reaching a value of 1 g/L and 2 g/L at 35 and 45 °C respectively, and thereafter its concentration dropped as a consequence of biogas production. Instead, butyric acid was obtained at the middle and toward the end of the experimental time, and it showed a high concentration (6.2 and 5.7 g/L at 35 and 45 °C respectively) regardless of biogas production. Under psychrophilic conditions (20 °C), VFAs production was extremely low.

The article "Bioengineering of anaerobic digestion for volatile fatty acids, hydrogen or methane production: A critical review" was retracted in 2026. Reason: compromised peer review.

Lee et al. [120] demonstrated how the choice of the optimal operative temperature is related to pH with respect to VFAs yields. They treated substrates in two different fermentation steps. The first one was at 55 °C without pH control. Under these conditions, the total VFAs production achieved was approximately 12 g/L. In the subsequent experimental run, the fermentation was carried out at 65 °C, both without pH control and set up at a pH value of 7.0. The VFAs production reached around 18 g/L with pH adjustment, a two-fold increment with respect to the experimental phase carried out under uncontrolled pH but slightly greater than the production achieved during the initial experimental phase at a lower temperature. Nevertheless, the temperature increase led to a good relative distribution of fermentation products, with acetic acid, propionic acid, and butyric acid accounting for the 39, 28 and 17%, respectively. A further increase of temperature until 70 °C, with the pH maintained at 7.0, brought to a higher total VFAs production of around 35 g/L. Under this condition, acetic acid was still the main fermentation product, accounting for 55% of total VFAs, but propionic acid was produced in lower amounts (14% of total production), while butyric acid was slightly more abundant, accounting for 31% of total VFAs obtained. A further increment of temperature until 80 °C led to a gradual decrease of VFAs production, up to a value similar to that obtained at 65 °C.

The article "Bioengineering of anaerobic digestion for volatile fatty acids, hydrogen or methane production: A critical review" was retracted in 2026. Reason: compromised peer review.

Therefore, it is clear that a higher working temperature, around thermophilic and hyperthermophilic range (up to 80 °C), leads to an increase of hydrolysis rate, giving hydroxylates theoretically available for fermentative microbial metabolism. Nevertheless, an increase of VFAs production is possible only according to optimal bacterial growing temperature, since many acidogens cannot survive at extreme temperature ranges [121].

#### 5.2.4. Hydraulic retention time (HRT)

Hydraulic retention time (HRT) can be defined as the average length of time that matter (both substrate and biomass) remains in a bioreactor. Consequently, it is an important parameter, especially in a full-scale perspective, since it establishes the flow rate treated in the bioreactor. It should be long enough to allow solubilization of complex organic matter thus favoring subsequent acidogenic fermentation of the hydrolyzates. At the same time, very long HRT reduces the quantity of substrate manageable per day and favors methanogens at suitable pH values. As many research on acidogenic food waste fermentation was carried out in batch bioreactors, little information is available in literature regarding the effect of HRT on overall VFAs production [122].

The appropriate retention time mainly depends on the type of substrate as it influences the hydrolysis rate. In some cases, however, the required retention time can differ with the same substrate (such as glucose). Therefore, the retention time does not only depend on the type of substrate but also on other operation conditions [123]. Jankowska et al. [123] observed that when HRTs of 5, 10, and 15 days were applied, the highest VFAs concentration was achieved after 15 days. Bolaji and Dionisi [124] applied HRTs of 10, 20, and 30 days for the anaerobic fermentation of vegetable and salad waste. Their results showed that an increase in HRT resulted in better VS reduction. Also, they detected the production of caproate after 20 and 30 days, although the main products were butyrate and acetate. Their results suggested that retention time influences not only the VFAs yield but also the product spectrum.

## 6. Composition of VFAs

The pH level plays a key role in determining the performance of the process, including the composition of VFAs produced. Feng et al. [22] studied the evolution of fermentation products and the changes in the microbial community along with pH variation using four long-term bioreactors and provided a detailed figure of the possible pathways. In summary, their report suggested that at pH 4.5–5.0, lactic acid and acetic acid were produced while pH 3.2–5.0 led to the biosynthesis of lactic acid, acetic acid and ethanol. In addition, it was proposed that glycolysis took place at pH 3.2–6.0 and that ethanol was produced at pH 4.4–6.0. At pH 3.2–6.0, the pentose phosphate metabolic pathway was established. At pH 6.0, acetic acid, butyric acid, valeric acid, acetone, ethanol, butanol, hydrogen, and carbon dioxide were produced with propionic acid and lactic acid being mostly converted into valeric acid. Lactic fermentation dominated due to the abundance of *Lactobacillus* at pH 3.2–4.5, reaching concentration of up to 13.5 g/L. On the other hand, *Bifidobacteria* increased significantly at pH 4.5, resulting in an increase of acetic acid. Butyric acid fermentation was observed at pH 4.7–5.0. *Bifidobacterium, Lactobacillus*, and *Olsenella* were still dominant at these conditions, but the lactic acid produced by them was rapidly converted to VFAs by microbes such as *Megasphaera, Caproicproducens* and *Solobacteria*. Mixed acid fermentation occurred at pH 6.0, with the highest VFAs concentration of 14.2 g/L, and the dominant microoganisms were *Prevotella* and *Megasphaera*. It was also observed that pH 4.5 and 4.7 led to the highest hydrolysis rate of 50% and an acidification rate of 45%.

The article "Bioengineering of anaerobic digestion for volatile fatty acids, hydrogen or methane production: A critical review" was retracted in 2026. Reason: compromised peer review.

The microbial performance toward diverse carboxylic acids by mixed bacterial communities utilizing heterogeneous waste streams, however, appears to be dependent on a combination of several factors. Some authors have provided contradicting accounts that suggest that the consideration of these factors in isolation might not be conclusive. For example, while operating at pH 3.9 ± 0.3 in a semi-continuous mode, Wainaina et al. [17] observed that the predominant metabolite from acidification of food waste was caproic acid unlike Wang et al. [4] who obtained mainly acetic acid using a similar substrate and pH conditions in batch bioreactors. During the biodegradation of food waste in alkaline conditions, Cheah et al. [125] reported acetate as the main VFA produced while Stein et al. [126] observed the highest yield of butyrate. In addition to the variations of the enriched microorganisms, these conflicting observations might be attributed to the disparities in the proportions of individual molecules, such as carbohydrates, proteins and lipids, in addition to other operating conditions such as the OLR and the HRT [98,127]. The changes in temperature can also influence the biosynthesis of VFAs from wastes. Stein et al. [126] and Jiang et al. [113] observed that the microbial productivity shifted from acetate to butyrate from food waste when the temperature was raised from 35 to 55°C. In another study using food waste, it was found that acetate took the largest share at 35 and 45°C, while propionate dominated at 25°C [98]. However, when waste activated sludge was used, the major metabolite was acetate at a wide range of 24.6, 35, 45, 50, 60 and 65°C [128]. Regarding the VFAs yield, fermentation of sludge at 55°C performed better compared to 35°C [128,129], while different results were obtained with food waste, that is, 45 > 35 > 55°C [113] and 35 > 45 > 25°C [98].

The article "Bioengineering of anaerobic digestion for volatile fatty acids, hydrogen or methane production: A critical review" was retracted in 2026. Reason: compromised peer review.

Taken together, the composition of VFAs is dependent not only on the initial inoculum seeded in the bioreactors but also on the various physicochemical parameters that contribute to microbial dynamics. Since the product profile during acidification can be a consequence of a blend of several parameters, the behavior of microbial performance for specific bioproducts requires extensive optimization steps. As demonstrated by Stein et al. [126], it is also possible to synthesize specific carboxylates at high yield from mixed culture fermentation. Design and implementation of such processes would ensure supply of high-value molecules with minimal purification requirements since minor amounts of other metabolites would be produced.

## 7. Strategies to minimize consumption of VFAs and hydrogen

In the conventional anaerobic digestion process, VFAs and hydrogen serve as precursors for production of biogas. The utilization of VFAs begins with their conversion, alongside carbon dioxide and hydrogen, into acetic acid via anaerobic oxidation facilitated by acetogens such as *Clostridium aceticum* and *Moorella thermoacetica* [130,131]. The enriched methanogenic archaea, made up of the acetotrophic (aceticlastic) and hydrogenotrophic groups, thereafter reduce the acetogenic products into methane and carbon dioxide [132]. Selective inhibition of methanogens in the microbial consortium is therefore vital to minimize the depletion of VFAs and hydrogen in the bioreactor, and some of the inhibition strategies are described below.

### 7.1. Acidic or alkaline pH

The pH level is one of the key parameters that considerably influence the rate of growth of the microbes involved in the AD process. For instance, the methanogenic archaea are most active at pH 7.0, and fairly active around pH 6.5–8.2 [133]. However, hydrolytic and acidogenic bacteria can be cultivated optimally at pH levels between 5.5–6.5, although a wider range from as low as pH 4.0 to as high as 11.0, depending on the substrate, can be employed [17,133–136]. Therefore, adjusting the pH toward certain acidic and alkaline regions can effectively inhibit methanogens, thereby promoting the accumulation of VFAs. An acidic microenvironment may be as a result of the increasing concentration of the organic acids in the bioreactor, which could lower the buffering capacity in the bioreactor. The overload of VFAs would then disrupt the balance of the AD reactions, resulting in suppression of the methanogens [136]. It is worth noting that at high organic loading, acetic acid largely affects aceticlastic methanogens compared to the hydrogenotrophic methanogens [135].

The article "Bioengineering of anaerobic digestion for volatile fatty acids, hydrogen or methane production: A critical review" was retracted in 2026. Reason: compromised peer review.

It however appears that acidic conditions are more favorable for production of VFAs from more easily degradable materials such as sorted food wastes compared to more complex biowastes such as sewage sludge. Alternatively, alkaline conditions have been applied for inhibition of methanogens and during the production of VFAs from sewage sludge [137–139]. This is coupled with the beneficial hydrolytic capabilities for proteins and carbohydrates in the sludge as well as improved sludge dewaterbility [140,141]. The enhanced solubilization of organics from sludge consequently improves the VFAs synthesis with numerous researchers suggesting that an optimum pH value of 10.0 [21,141–143]. However, from the literature observed, the treatment of the chemical-laden effluent from the acidification bioreactor was not considered. Moreover, the cost-effectiveness of the operating extreme acidic and alkaline conditions due to the use of reagents needed to adjust the pH levels need to be studied, especially in large-scale processes. Therefore, techno-economic analysis is needed to reveal the feasibility of such processes.

### 7.2. High OLR at short HRT

The conversion of organic waste into biogas largely depends on balanced rates of reaction involved in the different phases of anaerobic digestion. Moreover, thermodynamically viable carbon flow is based on the cooperation between the diverse sets of microbes in the microbial community [144]. At high OLR, a condition known as overloading, acidification of the bioreactor occurs as a result of the high accumulation of VFAs. The methanogenic archaea are then unable to effectively consume the VFAs as rapidly as they are being formed. This imbalance leads to further accumulation of VFAs and the inhibition of methanogens that is mainly caused by the severe pH decrease [135,145]. The impact of high organic loading rate on the anaerobic digestion process can be complemented by operating at short HRT in continuous (or semi-continuous) cultures. The HRT is the inverse of the dilution rate (D), which in turn is directly proportional to the maximum microbial growth rate (μ_max_). Fast-growing microbes can be actively sustained in the bioreactor at high dilution rates or short HRTs [146,147]. However, approximately 8–20 days are required as the minimum retention time for methanogens [77] and thus operating at shorter HRT would drastically wash out this group of microbes.

The article "Bioengineering of anaerobic digestion for volatile fatty acids, hydrogen or methane production: A critical review" was retracted in 2026. Reason: compromised peer review.

Operating at high OLR at short HRT might be a simple methane-inhibiting strategy that could also potentially result in a higher concentration of VFAs coupled with an increased volume reduction of solid organic wastes. Nevertheless, the likely consequence of such a strategy would be a high surge of undigested solids in the bioreactor caused by insufficient hydrolysis. This would minimize the access of the biocatalysts to the available nutrients due to low mass transfer. Tolerable organic loading and retention times should, therefore, be considered. In addition, strategies such as constantly draining the bioreactor to maintain acceptable amounts of suspended solids should be applied.

### 7.3. Chemical methane inhibitors

Methane-forming archaea can also be selectively deactivated by means of chemical inhibition. The most commonly used inhibitors are coenzyme M analogs such as lumazine, 2-bromoethanesulfonate (BES) and 2-mercaptoethanesulfonate (MES). Unlike other fermentative microbes applied for anaerobic digestion, methanogens consist of a cofactor known as coenzyme M that carries the methyl group usually reduced to methane by the help of methyl-CoM reductase. The coenzyme M analogs act as competitive inhibitors of the methyl transfer reaction at varying concentrations (between 5–50 mM) [148]. Other chemicals that have been successfully applied for the inhibition process include β-cyclodextrin (β-CD), propynoic acid, chloroform, and fluoroacetate [148–150].

The chemicals described above, however, might also affect the other microbes responsible for the biosynthesis of VFAs or hydrogen. For instance, some reports have proposed that other hydrogen-producing microbes, as well as acetogens, can potentially be altered by the addition of BES, in addition to the extra purchase cost [147,148]. Future studies could, therefore, study the inhibition mechanism on acidogens by the mentioned chemicals and possibly define the optimum chemical concentrations that would allow a stable performance of acidification bioreactors.

### 7.4. Heat shocking of microbial consortium

The capability of acidogens to form spores when subjected to extreme conditions, such as high temperature, can be employed to deactivate the methanogenic microbes which lack the mentioned functionality. Valdez-Vazquez and Poggi-Varaldo [146] and Setlow [151] provided excellent descriptions of the sporulation mechanism. In summary, acidogens, belonging to the genera such as *Bacillus* and *Clostridium* responsible for biosynthesis of VFAs and hydrogen, can metabolically form spores that are resilient to heat shocking. Three distinct stages are involved in the sporulation process. Sudden rise in the temperature, up to 100°C for 15–120 min, activates the present spores in the acidogenic bacteria while vegetative cells in the inoculum are destroyed. The spores are largely dormant and are incapable of metabolic activity. The contact of the activated spore with certain germinant, such as L-alanine, L-asparagine, and L-valine, induces the second stage generally regarded as germination. New growing cells are then formed in the final stage of outgrowth [146,151,152].

The article "Bioengineering of anaerobic digestion for volatile fatty acids, hydrogen or methane production: A critical review" was retracted in 2026. Reason: compromised peer review.

It is, however, worth noting that the methane-forming archaea can survive the heat-shocking procedure if sufficient magnitude and exposure time are not provided [153]. This suggests that the effectiveness of the heat shock is dependent on the duration and the applied temperature. Future research could, therefore, be conducted to determine the optimal conditions, which can be supplied to prevent the flow of VFAs to the final phase of the anaerobic digestion process without excessive energy demand.

## 8. Volatile fatty acids recovery and purification

As stated earlier, the undissociated carboxylate species have the capacity to infiltrate the microbe’s cytoplasm and deprotonate inside the cell, thereby reducing the microbial performance. Furthermore, the biosynthesized VFAs from anaerobic digestion of wastes remain dissolved in solution, unlike biogas or hydrogen that can be collected from the bioreactor headspace. It is therefore critical to extract the VFAs to provide the favorable microenvironment by circumventing product inhibition as well as to supply the metabolites for further bioprocessing, purification or immediate application. The complexity of the recovery and/or purification method depends on the purposes mentioned above and can be carried out during (*in-situ*) or after the microbial degradation process (downstream). Compared to product recovery, purification is more intricate and involves concentrating the VFAs or fractionation of the individual metabolites. These processes can be carried out using membrane-based or chemical methods, with the former methods minimizing the exposure of the microbes to potentially harmful substances, and are discussed below.

### 8.1. In-situ extraction and purification

The *in-situ* extraction of VFAs from the anaerobic digestion medium can either be carried out continuously or intermittently without stopping the fermentation process. The potential of *in-situ* extraction processes for improving microbial activity due to reduced acid-related inhibition was reported by Nomura et al. [154] in which acetic acid was continuously removed during fermentation using *Acetobacter aceti*. The acid removal was associated with enhanced cell growth and higher productivity of up to 2.4 times greater compared to the system without the acid removal. This was achieved through electrodialysis, which is a procedure utilizing ion perm selective membranes to isolate charged ions in a solution when a voltage difference is created between two electrodes via electrolysis and dialysis principles [155]. Additionally, by decreasing the acetic and butyric acid concentrations, this separation technique has been found effective during hydrogen production bioreactors using sucrose and grass pellets as substrates [156].

The article "Bioengineering of anaerobic digestion for volatile fatty acids, hydrogen or methane production: A critical review" was retracted in 2026. Reason: compromised peer review.

Other promising extraction techniques involve incorporating pressure-driven membrane separation, such as microfiltration and ultrafiltration [17,140]. This can be achieved through immersed membrane panels or externally fitted modules. The major benefits of the mentioned processes are the low energy required to provide the driving force of the separation and the ease of integrating the membrane units with the anaerobic digestion systems. Moreover, such systems ensure high cell density in the bioreactors even at low HRTs, thereby promoting the microbial conversion process. However, these membrane-assisted recovery methods require strategies to reduce the imminent fouling caused by suspended materials in the fermentation medium, such as the cell biomass and organic nutrients, to ensure extended operation. The recovered solution rich in VFAs can be readily applied, for instance, to remove nitrogen and phosphorus from wastewater [140].

### 8.2. Downstream extraction and purification

The downstream procedures usually require the fermentation process to be halted. The procedures could also be performed as an additional step to the *in-situ* extraction described earlier in order to isolate particular carboxylates or remove the water content. This can be achieved through adsorption, which is a separation procedure dependent on the acids’ interaction with the applied adsorbent [157]. After adsorption, a desorption procedure is performed and then the adsorbent is regenerated for subsequent reuse. Different adsorbents, such as activated carbon and a variety of resins, possess different selective capacities for desired components [158]. It has previously been observed that the affinity of these absorbents on the acids is highly influenced by the carbon chain length; the longer the carbon chain, the better the adsorption performance [158,159]. Elsewhere, separation and concentration of VFAs produced from olive mill wastewater were performed using electrodialysis [155]. According to the authors, the recovered acids were poised to provide the carbon source for synthesizing polyhydroxyalkanoates (PHAs). In another research, a microbial bipolar electrodialysis cell achieved a VFAs recovery efficiency of 98.3% from the fermentation medium. The factors that influenced the VFAs recovery included the initial VFAs concentrations and composition as well as the applied voltage [160].

The article "Bioengineering of anaerobic digestion for volatile fatty acids, hydrogen or methane production: A critical review" was retracted in 2026. Reason: compromised peer review.

Other advanced pressure-driven membrane separation techniques have also been proposed. For instance, Zacharof and Lovitt [35] demonstrated a two-stage membrane, by combining ultrafiltration and nanofiltration processes, for the recovery of VFAs from the effluent from the anaerobic digestion of cattle slurry. The acid rejection efficiency during nanofiltration is directly related to the pH value and higher efficiency is achieved at values above the acid’s dissociation constant (pKa) than in lower pH values. Reverse osmosis by means of tight membranes under high pressure can also be used for VFAs isolation. For instance, Zhou et al. [161] showed that a reverse osmosis process could be applied optimally at 40°C, pH 2.9 and 20 bar to recover acetic acid. Another emerging VFAs separation technique is pervaporation, which is conducted by creating a concentration gradient across a membrane. It has been found to be effective for acid-water blends containing distinct components with close boiling points or that form an azeotrope [162]. During pervaporation, the membrane absorbs the compound with high affinity toward it and desorbs it on the permeate side in the form of vapor [163]. Successful separation of acetic acid was reported when poly (dimethylsiloxane) – and polybutadiene-based membranes were used [162].

## 9. Conclusion and future prospects

The preceding sections of this paper have provided a description of how the AD process can be employed for the production of intermediate metabolites with high market value, namely VFAs and hydrogen, instead of biogas. The high availability of organic wastes and residues, emanating from industries, municipalities, and agricultural activities, makes AD a sustainable avenue for the biosynthesis of these metabolites. Due to the vast application potentials of these intermediate products, it is envisioned that existing AD facilities would possibly be converted into biorefineries. This would, however, require appropriate modification of the microbial pathways in such a way that the reactions leading to their formation are enhanced. One other important factor for successful VFAs and hydrogen production is the termination of methanogens’ activities to prevent their flow to the last stage where they would be consumed.

The article "Bioengineering of anaerobic digestion for volatile fatty acids, hydrogen or methane production: A critical review" was retracted in 2026. Reason: compromised peer review.

The AD process employs undefined mixed culture systems that are robust and easy to handle relative to pure culture fermentations. In order to enhance the biosynthesis of VFAs from AD systems, several operational factors, including the applied temperature, pH, OLR, and HRT, should be optimized. It should also be noted that the interaction of these factors might exist and that the process might also be influenced by the molecular composition of the substrate used. Moreover, the diversity in the microbes enriched in the AD bioreactor usually results in a mixture of VFAs and other secondary products. Therefore, the development of new microbial consortia for greater productivity is an urgent necessity because single microbes are not capable of utilizing all kinds of substrates for the production of VFAs and require costly operating conditions. In this regard, the evolutionary bioengineering and new metagenomic techniques could be beneficial to improve the tolerance of developed microbial consortium and enhance VFAs productivity.

Prior to the fermentation process, difficult-to-degrade organic wastes need to be disintegrated to allow for microbial access to the available nutrients. The accumulated carboxylates could easily penetrate into the cell and potentially reduce the microbial performance. Removal of the accumulated VFAs during fermentation, using for instance membrane-assisted methods, helps to prolong the microbes’ activity and provides utilizable VFAs-rich product streams. The recovered VFAs can be immediately applied for replacing fossil-derived carbon sources in processes such as the removal of nutrients in wastewater treatment plants. Other important factors that require further research attention include optimization of bioreactor designs and development of sustainable techniques to enhance product purity for industrial implementation. The fractionated acids can potentially be used in essential areas such as in the food and pharmaceutical industries.

## Highlights

- The anaerobic digestion process can be manipulated to produce high-value products
- This paper explains the theory of acidogenic reactions within anaerobic digestion
- The acidogenic reactions result in production of VFAs and hydrogen
- Inhibition of methanogens is key for accumulation of VFAs and hydrogen
- Favorable microenvironment for acidogens is enabled by *in-situ* product recovery
